The article "G Protein Subunit Gamma 5 Is a Prognostic Biomarker and Correlated with Immune Infiltrates in Hepatocellular Carcinoma" was retracted in 2023. Reasons: signs of a paper mill; suspected computer-generated content; unreliable results or conclusions; concerns about the data.

# G Protein Subunit Gamma 5 Is a Prognostic Biomarker and Correlated with Immune Infiltrates in Hepatocellular Carcinoma

**DOI:** 10.1155/2022/1313359

**Published:** 2022-05-31

**Authors:** Hang Wang, Liang Yu, Yunfu Cui, Jiaxin Huang

**Affiliations:** ^1^Department of Hepatopancreatobiliary Surgery, Second Affiliated Hospital of Harbin Medical University, Harbin 150086, China; ^2^The Key Laboratory of Myocardial Ischemia, Harbin Medical University, Ministry of Education, Harbin 150086, China; ^3^Department of Pathology, Li Ka Shing Faculty of Medicine, The University of Hong Kong, Hong Kong; ^4^Department of Postgraduate, Third Affiliated Hospital of Harbin Medical University, Harbin Medical University, Harbin 150081, China

## Abstract

Hepatocellular carcinoma (HCC) is one of the malignancies with an extremely inferior prognosis in the abdominal cavity, making it essential to develop more effective biomarkers for HCC. Although GNG5 has been linked to increased patient survival in a variety of human malignancies, no evidence has been found for its involvement in the development of HCC yet. Our study first analyzed the expression and prognosis of GNG5 in HCC using The Cancer Genome Atlas database (TCGA database) with the Gene Expression Omnibus database (GEO database) and found that GNG5 has a potential oncogenic role. Based on survival analysis, the clinical importance and prognostic value of the GNG5 gene were studied. Relying on tumor Immune Estimation Resource database (TIMER database), we analyzed the correlation between the GNG5 gene and HCC Immune infiltration cells. GNG5 expression levels were significantly higher in HCC tissues compared to normal liver tissues. HCC patients with high GNG5 expression had significantly reduced overall survival time and affected multiple immune cell infiltrates. Additionally, KEGG functional enrichment analysis indicated the PI3K-Akt signaling pathway as the most promising carcinogenic pathway associated with GNG5. This is the first comprehensive revelation of GNG5 as a possible new biological marker associated with immune infiltration in HCC. Additionally, it holds promise as an emerging target for HCC immunotherapy.

## 1. Introduction

Hepatocellular carcinoma (HCC) represents one of the most common malignancies worldwide, accounting for the third highest number of cancer-related fatalities. Every year, more than 750,000 new cases are diagnosed, with a 5-year survival rate of only 11% [1]. Although studies of prognostic risk factors for HCC have proliferated in recent past, such as viral infections [2], cirrhosis [3], alcohol [4] abuse, and immune system disorders [5], However, the trend of HCC patients' morbidity still cannot be curbed, while most patients are diagnosed with advanced tumors. To date, surgical resection remains the primary means of tumor reduction in the treatment of patients with HCC [6]. The 5-year survival rate for patients undergoing surgical treatment is 30-50% [7], but such prognosis remains unsatisfactory. Recent studies have found that the immune microenvironment performs a soil-like character in the development of tumors as well as in cancer treatment [8]. According to the theory of immune microenvironment, tumor cells do not grow in isolation but interact with other cells such as surrounding endothelial cells and fibroblast immune cells, leading to macrophage infiltration and fibroblast proliferation and angiogenesis, which together determine the progression of the tumor [9]. Immunotherapy for liver cancer, represented by immune checkpoint inhibitors, is being used in conjunction with traditional HCC treatments to further improve patient prognosis [10].

It is known that the G protein subunit Gamma 5 (GNG5), a member of the G protein family, plays a role in many cellular functions, including cell division, differentiation, and metastasis, during embryonic development [11]. GNG5 has been implicated in glioma progression and invasion [12]. Over the last decade, aberrant expression of other G-protein family members has been involved in oncogenesis, including gastric cancer [13], renal clear cell carcinoma [14], esophageal cancer, and colorectal Cancer [15]. However, the expression of GNG5 in hepatocellular carcinoma and its prognostic value have not been reported.

The purpose of this article is to shed light on the utility of GNG5 in predicting prognosis in hepatocellular carcinoma and its association with immune cell infiltration and immune checkpoints. In bioinformatics, it helps to demonstrate that GNG5 can be used as a biological marker in hepatocellular carcinoma, thus providing a strategy to study the role of immune-related genes in hepatocellular carcinoma.

## 2. Material and Methods

### 2.1. Database and Information Collection

The Cancer Genome Atlas (TCGA) (visit website: http://portal.gdc.cancer.gov/) contains clinical data of various human cancers, mRNA, and other data. It is an important source of data for cancer researchers. Gene expression data and medical characteristic information of HCC patients were collected from the TCGA database, which included 374 hepatocellular carcinoma tissue samples and 50 normal liver tissue samples. We further collected 110 normal liver tissue samples from the GTEx database (visit website: http://www.gtexportal.org/home) as a control group. In addition to further evaluate the accuracy of GNG5 gene expression in predicting the prognosis of HCC patients, we collected RNA sequencing data and corresponding clinical information from the ICGC database (visit website: http://dcc.icgc.org/) for 232 HCC patients. This part of the data served as a validation dataset for the prognostic risk model. The UALCAN database (visit website: http://ualcan.path.uab.edu/index.html) is our main database for obtaining protein expression levels of GNG5 and corresponding clinical information; we also used the HPA database (visit website: http://www.proteinatlas.org/) to obtain GNG5 in HCC tissues immunohistochemical results. Paired normal liver tissues with liver cancer tissues were from the same patient (Patient id: 2279) in the HPA database. Image results from conventional immunohistochemistry by applying antibodies (Atlas Antibodies Cat#HPA043651).

### 2.2. Construction and Validation of Clinical Prognostic Models

All HCC patient information was obtained from the TCGA database. Selected patients were treated in accordance with the AASLD Guidelines for the Treatment of Hepatocellular Carcinoma. All patients older than 18 years of age and diagnosed with HCC were screened into our study. The data of 374 cases were classified into GNG5 high-expressing level group and low-expressing level group. Cut-off value is the median expression of GNG5. Information on patient characteristics is shown in Table 1. Kaplan-Meier curves were plotted to compare overall survival (OS) differences, and time-dependent ROC curves were used to compare prediction accuracy. Prognostic risk factors were determined using univariate Cox proportional risk regression and multivariate Cox proportional risk regression, using ggplot 2 and the survival R package to generate nomograms and plot calibration curves.

### 2.3. Analysis of Differentially Expressed Genes and Functional Enrichment Analysis

We used HCC tumor tissues from the TCGA database with normal tissue samples from the GTEx database for further analysis. Differential expression gene was achieved using DESeq2 R package. The criteria for discovering DEGs were as follows: (1) adjusted *P* < 0.05 and (2) |Log2FC| ≥ 1.5. Enrichment analysis was performed using the ClusterProfiler R package, including Gene Ontology (GO) and the Kyoto Encyclopedia of Genes and Genomes (KEGG). For the enrichment results, an adjusted *P* < 0.05 was considered significant.

### 2.4. Immune Infiltration Analysis

We analyzed the infiltration of immune cells in tumor tissues for specific RNA-Seq expression profile data using the TIMER database (https://cistrome.shinyapps.io/timer/). The abundance of different immune cells between the high and low GNG5 expression groups was assessed by the CIBERSORT algorithm, and *P* < 0.05 was considered statistically significant. T Immune checkpoint analysis and immune correlation score analysis were plotted applying the ggplot2 R package.

### 2.5. Drug Sensitivity Analysis

Using the pRRophetic R package, the minimal drug inhibitory concentrations (IC50) of antitumor drugs were analyzed in HCC patients in the GNG5 high and low expression groups.

### 2.6. Statistical Methods

All statistical analyses were run in the R (v.4.1.2) software as well as in the Statistical Package for Social Science Software (version 24.0; IBM Corporation). A *t*-test was used for differences between groups; Pearson's or Spearman's correlation test was used for correlation analysis. We used overall survival as the focus event of the study. Kaplan-Meier curves were used to estimate OS in different groups, and differences between curves were analyzed by a log-rank test. Univariate and multivariate Cox regression models were used to estimate hazard ratios (HR) and 95% confidence intervals (CI), and *P* values < 0.05 were considered statistically significant.

## 3. Results

### 3.1. Expression Level of GNG5 in Hepatocellular Carcinoma

The GNG5 gene may have similar effects in different human cancers. Therefore, we first observe the expression in GNG5 in different human cancers. Combining the database information of TCGA and GTEx for analysis, we found that the mRNA levels of GNG5 were upregulated in most cancers; these include hepatocellular carcinoma, bile duct cancer, colon cancer, lung cancer, pancreatic cancer, gastric cancer, thyroid cancer, adrenocortical cancer, prostate cancer, and breast cancer. However, expressions of GNG5 in Kidney Chromophobe and Acute Myeloid Leukemia were downregulated (Figure 1(a)). In different databases, GNG5 was present at higher expression levels in HCC tissues comparing to normal tissues (*P* < 0.001) (Figures 1(b) and 1(c)). The results showed that the expression levels of GNG5 were elevated in HCC tissues of different histological grade, pathological stage, T-stage, age group, and gender compared to normal patients (each *P* < 0.01) (Figures 1(d)–1(h)).

### 3.2. Elevated Expression of GNG5 Protein in Hepatocellular Carcinoma

Our study further analyzed the expression of GNG5 protein in HCC tissues. Derived from the UALCAN online tumor database, we observed that the expression level of GNG5 protein was significantly elevated in HCC tumor tissues (Figure 2(a)). This phenomenon also occurred in tumor tissues of patients of different sexes and ages (Figures 2(b) and 2(c)). According to the images of immunohistochemical results of paired tissues from patients with hepatocellular carcinoma in the HPA database, GNG5 became strongly positive in HCC tissues, while it became medium colored in normal liver tissues. Therefore, immunohistochemical results of clinical HCC samples also observed significantly higher levels of GNG5 in the tumor tissue than in the adjacent normal liver tissue (Figures 2(d) and 2(e)).

### 3.3. Functional Prediction of GNG5 in HCC

The study of differentially expressed genes (DEGs) is essential if we are to explore the mechanisms of tumorigenesis and potential biological roles of genes. We used data from the TCGA transcriptome for our analysis. We observed 1146 DEGs associated with GNG5 gene expression. To visualize the results, we constructed a volcano plot of 977 upregulated and 169 downregulated DEGs (Figure 3(a)); the heatmap shows the first five up- and downregulated DEGs (Figure 3(b)). To more visualize the function of 1146 DEGs associated with GNG5 expression in hepatocellular carcinoma. In this study, GO and KEGG functional enrichment indicated that most of these genes were involved in the following events: association with biological processes (BP) including extracellular matrix, extracellular structures and external envelope structures; cellular components (CC) including extracellular matrix, collagen trimer, and endoplasmic reticulum lumen; and molecular function (MF) including extracellular matrix structural constituent, glycosaminoglycan binding, and heparin binding. KEGG analysis was associated with PI3K-Akt signal pathway, focal adhesion, and neuroactive ligands and receptor pathway.

### 3.4. The Value of GNG5 as a Biological Indicator of HCC Prognosis

To investigate whether GNG5 expression correlates with the prognosis of HCC patients, we evaluated the correlation among the expression levels of GNG5 and patient survival using the TCGA and ICGC databases. We divided the patient records into the high expression and low expression groups according to the median GNG5 expression. Based on Kaplan-Meier survival curves, we found that an elevated expression of GNG5 tended to be correlated with poor survival time in HCC (*P* = 0.00372) (Figure 4(b)). We further plotted time-dependent ROC curves for GNG5 predicting 1-, 3-, and 5-year survival, with AUC values above 0.6 (Figure 4(c)). For such results, we did a validation analysis using the ICGC database. The results showed that GNG5 expression was associated with poorer survival time (*P* = 0.0409) (Figure 5(b)). The AUC values of the time-dependent ROC curves at 1, 3, and 5 years were all above 0.6 also indicated a predictive role of GNG5 (Figure 5(c)). Taken together, these consistent results of OS analysis suggest the great value of GNG5 as a biological marker for predicting the prognosis of HCC patients.

### 3.5. GNG5 Combined with Clinical Characteristic Factors to Predict Prognosis of HCC Patients

To more accurately predict the survival time of HCC patients, we used the expression of GNG5 in combination with other clinical characteristic factors to predict the prognosis of patients. Clinical characteristic factors such as age, gender, T-stage, TNM classification, and pathological grade were considered into this study. The forest plot demonstrates that GNG5 expression, staging, and TNM classification were all considered as risk factors affecting the prognosis of HCC patients after using univariate Cox regression (Figure 6(a)). After multivariate Cox proportional risk regression assessment, GNG5 (*P* = 0.00114) with T-stage (*P* = 0.00001) was identified as a risk factor in the prognostic model (Figure 6(b)). The RMS R package was used to construct the OS nomogram (Figure 7(a)). In clinical practice, we can use this nomogram to accurately calculate the risk of 1-, 3-, and 5-year survival times for HCC patients. According to the nomogram calibration curve, the prediction results of this model were highly consistent with the observation of all patients (Figure 7(b)).

### 3.6. Correlation of GNG5 Expression with Immune Characteristics

To explore the correlation between GNG5 expression and immune characteristics, we did Spearman's correlation analysis using the expression of GNG5 in the tumor microenvironment and the level of immune cell infiltration, and the results showed that GNG5 was positively correlated with Th2 cells, TFH, macrophages, aDC, Th1 cells, T cells, helper T cells, iDC, NK CD56bright cells, and B cells; positively correlated with Th17 cells and Tcm cells; negatively correlated with Th17 cells and Tcm cells (Figure 8(a)). Immune score (*r* = 0.244, *P* < 0.001), stromal score (*r* = 0.078, *P* = 0.132), and ESTIMATE score (*r* = 0.190, *P* < 0.001) were associated with HCC. All were positively correlated with the expression of GNG5 (Figure 8(b)). Our study also observed multiple immunotherapeutic targets, including CD247, PDCD1, CTLA-4, LAG3, HAVCR2, PDCD1LG2, and TIGIT, were significantly positively associated with expressions of GNG5 (Figures 9(a)–9(g)).

### 3.7. Correlation of GNG5 Expression with Immune Infiltrating Cells in HCC Patients

We speculated whether the expression of GNG5 could influence HCC immune infiltration. To confirm our hypothesis, we analyzed the correlation between GNG5 expression and immune cell biomarkers using the TIMER database. As shown in Table 2, we observed that GNG5 expression was positively correlated with the expression of many immune cell biomarkers. These immune markers include B cells (CD19, CD20, and CD38), CD8+ T cells (CD8A and CD8B), M1 macrophages (IRF5 and PTGS2), M2 macrophages (CD115 and CD206), TAM (PDCD1LG2, CD80, CD40, and TLR7), natural killer cells (CD7 and XCL1), neutrophils (ITGAM, CEACAM8, and FUT4), and dendritic cells (CD1C, THBD, and ITGAX) and other T cell subset biomarkers.

### 3.8. Analysis of Sensitivity Difference of Antitumor Drugs in Different Groups

Since high expression of GNG5 has an extremely poor prognostic impact on HCC and to guide the sensitivity of HCC patients to antitumor drugs. We analyzed the IC50 differences between the GNG5 high and low expression groups for sensitivity to different antitumor drugs. The GNG5 high expression group was found to be more sensitive to QS11, paclitaxel, PAC-1, LFM-A13, OSU-03012, LAQ824, etoposide, AUY922, vinorelbine, and sunitinib which were more sensitive. This suggests the possibility that these antitumor agents are more effective in patients at high risk of HCC. This also provides new ideas for developing different treatment regimens in the clinic (Figures 10(a)–10(h)).

## 4. Discussion

The early diagnosis and treatment of hepatocellular carcinoma remain suboptimal. It is critical to identify more effective drug targets for HCC or to find promising biomarkers. Numerous studies have established that the G protein family is involved in the development and progression of a variety of human gastrointestinal cancers [16–18], including HCC [19]. To begin, we used The Cancer Genome Atlas (TCGA) database to conduct a pan-cancer analysis of GNG5 expression. The expression of GNG5 was found to be upregulated in numerous tumors. Then, we further verified the expression of GNG5 protein using the UALCAN database and obtained results consistent with gene expression. To investigate whether high GNG5 expression could affect the overall survival of HCC patients, we divided the GNG5 expression level into high and low expression groups. And it was observed that patients in the high GNG5 expression group had a significantly worse prognosis; this grouping could effectively distinguish the prognosis of patients. Our analysis of the relationship between clinical characteristics and prognosis of HCC patients revealed that GNG5 expression and T stage can be independent predictors of OS in HCC. This further enriches the applicability of GNG5 in clinical applications. A poor prognosis was found in HCC patients with high GNG5 expression, suggesting GNG5 could be a prognostic factor in hepatocellular carcinoma. Single biological markers are often poor predictors of patient prognosis [20], and we can also combine classical biological markers of HCC such as AFP to make judgments about the early diagnostic calculations and prognosis of patients.

Heterotrimeric (alpha-beta-gamma) G-proteins are membrane-associated proteins that directly bind to the G protein-coupled receptors (GPCRs) to contribute to signal transduction, dysregulation in either can fundamentally affect the inception of pathogenic cycles. To be sure, the practical jobs of G-proteins and GPCRs in inflammation, cell communication, and the variety of ligands they tie lay out both as significant controllers of the tumor-immune microenvironment [21, 22]. According to the TIMER database, our findings revealed a link between GNG5 expression and a variety of tumor-infiltrating immune cells. To be more specific, GNG5 was found to be linked to Th2 cells, TFH, macrophages, aDC, Th1 cells, T cells, T helper cells, iDC, NK CD56bright cells, and B cells. Furthermore, the immune score, stromal score, and ESTIMATE score of HCC were all significantly correlated with the expression of GNG5. In the tumor microenvironment, many factors influence the typical immune function of tumor-infiltrating immune cells. It was discovered that by producing growth factors, chemokines, stromal degrading enzymes, and supporting tumor cells, all components of the TME contribute to cancer proliferation and metastasis. Tumor suppressor factors secreted by cancer cells, stromal fibroblasts, and other cells in a complex tumor microenvironment (TME) play a critical role in current antitumor immunotherapy by suppressing the antitumor activity of immune cells and producing immunosuppressive effects, which play a critical role in poor prognosis and little improvement in the prognosis of patients. The potential value of GNG5 in HCC remains to be further explored. In this study, KEGG analysis showed that GNG5 is involved in the PI3K/Akt signaling pathway, suggesting that GNG5 may regulate the growth of HCC by activating the PI3K/Akt signaling pathway. PI3K activates its downstream molecule Akt, leading to phosphorylation and ultimately promoting tumor growth. This pathway has been reported to play a key role in many biological processes of tumors, such as proliferation, migration, and survival [23]. We also found that GNG5 is closely associated with cell adhesion and downregulation of GNG5 may inhibit HCC proliferation and migration through the cell adhesion molecule pathway. These findings provide new ideas and research prospects for GNG5 in the treatment of HCC.

For therapeutic aspects, we performed differential analysis of GNG5 expression with different antitumor agents and found that many chemotherapeutic agents or targeted agents may inhibit high-risk hepatocellular carcinoma at relatively small doses. We also found that gene expression of numerous promising immunotherapeutic targets (including CD247, PDCD1, CTLA-4, LAG3, HAVCR2, PDCD1LG2, and TIGIT) was significantly positively correlated with GNG5 expression. Additionally, GNG5 was associated with a variety of immune infiltrating cells (CD8+ T cells, T cell subsets, B cells, M1 macrophages, and TAM biomarkers, among others) which were significantly positively correlated with biomarkers. GNG5 may be able to have oncogenic effects via boosting tumor immune cell infiltration and the expression of immune checkpoints, as evidenced by these findings. It also provides a new feasible idea that targeting GNG5 may improve the immunotherapeutic effect of HCC. Immunotherapy for liver cancer, as represented by immune checkpoint inhibitors, has gradually resulted in a paradigm shift in the treatment of. For example, sintilimab in combination with a biosimilar bevacizumab (IBI305) can improve overall survival in Chinese patients with advanced HBV-related HCC when compared to sorafenib [24]. However, only 25% of HCC patients with infiltrated T cells expressing high levels of PD-1 were found responding to immune checkpoint inhibitor therapy [25]. It suggests that the key genes and mechanisms of the immune microenvironment of HCC are complex and need to be further explored. HCC patients who are sensitive to immunotherapy also need to be further identified for individualized treatment to improve the core treatment strategy for liver cancer patients. However, there are several limitations to this research. For example, the number of normal samples in the TCGA database is quite limited, and the theory has not been tested in cellular or animal models to determine its validity.

## 5. Conclusion

We verified the utility of GNG5 in the diagnostic and prognostic prediction of hepatocellular carcinoma in this study. Increased GNG5 expression was related with a worse outcome for hepatocellular carcinoma. GNG5 may be involved in the genesis and progression of HCC, as well as in the immunological modulation of the disease. Therefore, GNG5 may serve as a diagnostic and predictive biomarker for hepatocellular carcinoma, as well as a therapeutic target.

## Figures and Tables

**Figure 1:** (a) Differential expression levels of GNG5 in tumors versus normal tissues, based on TCGA and GTEx databases. (b) Protein levels of GNG5 were significantly elevated in hepatocellular carcinoma tissues of different genders compared to normal samples. (c) Protein levels of GNG5 were significantly elevated in hepatocellular carcinoma tissues of different age groups compared to normal samples (*P* < 0.001). (d–h) The association between the expression levels of GNG5 and clinical characteristics in HCC. It shows that GNG5 expression remained elevated in different clinical subgroups of histologic grade, pathologic grade, T stage, age, and gender.

**Figure 2:** Results of protein level expression of GNG5 in UALCAN and HPA databases. (a) Upregulation of GNG5 protein level expression in HCC tissues. (b) GNG5 protein levels are elevated in different sexes than in normal samples. (c) GNG5 protein levels were elevated in different age subgroups compared to normal samples. (d, e) Immunohistochemical results showed that the protein expression level of GNG5 was elevated in HCC tissues compared with normal liver tissues.

**Figure 3:** An analysis of DEGs between high and low GNG5 expression in TCGA-HCC patients. (a) A volcano map of differentially expressed genes shows 977 upregulated genes and 169 downregulated genes. (b) RNA heatmaps of 5 upregulated genes and 5 downregulated genes. (c, d) KEGG enrichment and GO enrichment analysis by GNG5 expression-correlated upregulation.

**Figure 4:** Results of TCGA dataset analysis: prognostic analysis of GNG5 expression levels on overall survival time of HCC. (a) Heatmap of GNG5 expression distribution, survival status and GNG5 expression profile. (b) Patients in the high GNG5 expression group had a significantly shorter overall survival time than the low GNG5 expression group. (c) Time-dependent ROC curve of GNG5 expression predicting prognostic risk of patients.

**Figure 5:** Results of ICGC validation dataset analysis: prognostic an0alysis of GNG5 expression levels on overall survival time of HCC. (a) Heatmap of GNG5 expression distribution, survival status and GNG5 expression profile. (b) Patients in the high GNG5 expression group had a significantly shorter overall survival time than the low GNG5 expression group. (c) Time-dependent ROC curve of GNG5 expression predicting prognostic risk of patients.

**Figure 6:** Risk analysis of GNG5 expression and other clinically characteristic factors affecting OS in HCC patients. (a) In univariate Cox regression analysis, GNG5 expression, T stage, and TNM classification were determined to have a statistically significant relationship with OS. (b) Expression of GNG5 and T-stage in multi-Cox regression analysis was the final clinical risk factor to predict OS in HCC.

**Figure 7:** Prognostic risk model for HCC was constructed. (a) Nomogram that can predict the 1-, 3-, and 5-year survival probability of HCC diagnosis. (b) Calibration curve of the prognostic risk model for HCC.

**Figure 8:** (a) Lollipop plot of the correlation between GNG5 expression and immune infiltrating cells. (b) GNG5 expression was significantly and positively correlated with immune score, stromal score, and ESTIMATE score.

**Figure 9:** Correlation of GNG5 expression with immune checkpoint expression in HCC (a) CD247, (b) PDCD1, (c) LAG3, (d) HAVCR2, (e) CTLA-4, (f) PDCD1LG2, and (g) TIGIT.

**Figure 10:** Differences in IC50 between the effects of antitumor drugs on GNG5 high and low expression groups. (a–j) Antitumor drugs such as QS11, paclitaxel, PAC-1, LFM-A13, OSU-03012, LAQ824, etoposide, AUY922, vinorelbine, and sunitinib showed higher drug sensitivity in the GNG5 high expression group.

**Table 1:** Characteristics information table of HCC patients.

Characteristic	Low expression of GNG5	High expression of GNG5	*P*
	187	187	
T stage, *n* (%)			0.217
T1	99 (26.7%)	84 (22.6%)	
T2	42 (11.3%)	53 (14.3%)	
T3	39 (10.5%)	41 (11.1%)	
T4	4 (1.1%)	9 (2.4%)	
N stage, *n* (%)			0.122
N0	127 (49.2%)	127 (49.2%)	
N1	0 (0%)	4 (1.6%)	
M stage, *n* (%)			1.000
M0	132 (48.5%)	136 (50%)	
M1	2 (0.7%)	2 (0.7%)	
Pathologic stage, *n* (%)			0.273
Stage I	96 (27.4%)	77 (22%)	
Stage II	39 (11.1%)	48 (13.7%)	
Stage III	39 (11.1%)	46 (13.1%)	
Stage IV	2 (0.6%)	3 (0.9%)	
Gender, *n* (%)			0.047
Female	51 (13.6%)	70 (18.7%)	
Male	136 (36.4%)	117 (31.3%)	
Age, *n* (%)			0.133
≤60	81 (21.7%)	96 (25.7%)	
>60	106 (28.4%)	90 (24.1%)	
Histologic grade, *n* (%)			0.002
G1	35 (9.5%)	20 (5.4%)	
G2	97 (26.3%)	81 (22%)	
G3	51 (13.8%)	73 (19.8%)	
G4	2 (0.5%)	10 (2.7%)	

**Table 2:** Correlation analysis between GNG5 expression and immune cell markers in HCC.

Immune cell	Biomarker	Cor	*P* value
B cell	CD19	0.307	<0.001
	CD20 (KRT20)	0.165	0.001
	CD38	0.323	<0.001
CD8+ T cell	CD8A	0.322	<0.001
	CD8B	0.336	<0.001
Tfh	BCL6	0.038	0.459
	ICOS	0.363	<0.001
	CXCR5	0.245	<0.001
Th1	T-bet (TBX21)	0.185	<0.001
	STAT1	0.339	<0.001
	STAT4	0.318	<0.001
	IL12RB2	0.128	0.013
	WSX1 (IL27RA)	0.313	<0.001
	IFN-*γ* (IFNG)	0.301	<0.001
	TNF-a (TNF)	0.274	<0.001
Th2	CCR3	0.23	<0.001
	GATA3	0.344	<0.001
	STAT5A	0.315	<0.001
	STAT6	0.049	0.34
Th9	IRF4	0.313	<0.001
	PU.1 (SPI1)	0.444	<0.001
	TGFBR2	-0.007	0.89
Th17	IL-17A	-0.056	0.277
	IL-21R	0.393	<0.001
	IL-23R	0.142	0.006
	STAT3	0.216	<0.001
Th22	AHR	-0.11	0.033
	CCR10	0.36	<0.001
Treg	CCR8	0.264	<0.001
	CD25 (IL2RA)	0.416	<0.001
	FOXP3	0.171	<0.001
M1 macrophage	COX2 (PTGS2)	0.235	<0.001
	INOS (NOS2)	0	0.993
	IRF5	0.211	<0.001
M2 macrophage	ARG1	-0.084	0.104
	CD206 (MRC1)	0.103	0.047
	CD115 (CSF1R)	0.349	<0.001
TAM	PDCD1LG2	0.224	<0.001
	CD80	0.383	<0.001
	CD40	0.211	<0.001
	TLR7	0.38	<0.001
Natural killer cell	CD7	0.374	<0.001
	KIR3DL1	0.023	0.657
	XCL1	0.371	<0.001
Neutrophil	CD11b (ITGAM)	0.306	<0.001
	CD15 (FUT4)	0.397	<0.001
	CD66b (CEACAM8)	0.113	0.028
Dendritic cell	CD1C	0.221	<0.001
	CD11c (ITGAX)	0.329	<0.001
	CD141 (THBD)	0.104	0.044

## Data Availability

The data that support the findings of this study were derived from the following resources available in the public domain: The Cancer Genome Atlas (http://portal.gdc.cancer.gov/), Genotype-Tissue Expression (http://gtexportal.org/home), International Cancer Genome Consortium (http://dcc.icgc.org/), and UALCAN (http://ualcan.path.uab.edu/index.html).
